The article "Investigation of the Effects of Large Bone Flap Craniotomy on Cerebral Hemodynamics, Intracranial Infection Rate, and Nerve Function in Patients with Severe Craniocerebral Trauma" was retracted in 2023. Reasons: signs of a paper mill; suspected computer-generated content; unreliable results or conclusions; lack of ethics approval or compliance.

# Investigation of the Effects of Large Bone Flap Craniotomy on Cerebral Hemodynamics, Intracranial Infection Rate, and Nerve Function in Patients with Severe Craniocerebral Trauma

**DOI:** 10.1155/2022/2681278

**Published:** 2022-09-02

**Authors:** JiNan Li, XinLi Zhang, Hang Su, YaNan Qu, Meixuan Piao

**Affiliations:** Affiliated Zhongshan Hospital of Dalian University, Dalian 116001, China

## Abstract

In order to explore the clinical value of large bone flap craniotomy, the effects of standard large bone flap craniotomy on cerebral hemodynamic indexes, incidence of postoperative intracranial infection, and neurological function in patients with severe craniocerebral trauma are investigated. 89 patients with severe craniocerebral trauma admitted from January 2020 to June 2021 are analyzed retrospectively. All patients are divided into a large craniotomy group (*n* = 45) and control group (*n* = 44) according to different surgical methods. The large craniotomy group is treated with large craniotomy decompression, and the control group is treated with traditional craniotomy decompression. The incidence of intracranial infection in each group is recorded, and NIHSS is applied to observe the neurological function recovery of 2 groups before and 1 month after operation. Besides, the patients are followed up after surgery and the Kaplan–Meier survival curve is obtained to compare the survival rate of patients in the two groups. It is clearly evident that the two surgical methods have certain clinical efficacy in the treatment of patients with severe craniocerebral trauma. Comparatively, the large craniotomy can further improve brain blood supply and improve neurological function recovery. Also, it can obtain low incidence of postoperative adverse reactions and intracranial infection.

## 1. Introduction

As one of neurosurgery common type of disease, severe craniocerebral injury often leads to the loss of nerve function, leading to serious disturbance of consciousness, hemiplegia, aphasia, seizures, and even long-term vegetative state. Most of the patients suffered from brain injury caused by external impact and traffic accidents, accompanied by mental disorder, severe concussion, sharp rise of intracranial pressure and other clinical symptoms, and the progress was rapid. It can cause skull base fracture, cerebrospinal fluid leakage, subarachnoid hemorrhage, subdural hemorrhage, primary brain stem injury, and diffuse axonal injury. Therefore, the disease has the characteristics of high mortality, which seriously threatens the life and health of patients [1]. According to incomplete statistics, the mortality of patients with severe craniocerebral injury can reach more than 50%. Although the patients can maintain their lives after operation, some patients still have severe coma and vegetative life and the survival prognosis is generally poor. They are one of the serious clinical diseases [2]. At present, surgical treatment is one of the most effective methods to control the progress of severe craniocerebral injury. Through surgical treatment, the intracranial pressure can be rapidly reduced, the focus can be cleared, and the prognosis of patients can be effectively improved [3]. Traditional craniotomy decompression is one of the widely used surgical methods for patients with severe craniocerebral injury. It can alleviate the clinical symptoms of patients to a certain extent, but the effect of reducing intracranial pressure is limited due to the large trauma. In other words, there are limitations in improving patient prognosis and survival [4]. With the continuous development of medical technology, large bone flap craniotomy has been gradually applied in clinical practice. Large bone flap craniotomy has the following advantages: (1) complete hemostasis, removal of necrotic tissue, and intracranial hematoma; (2) effective reduction of intracranial pressure; and (3) improvement of cerebral blood flow and cerebral oxygen partial pressure. It should be noted that the clinical efficacy of large bone flap surgery in the treatment of patients with severe craniocerebral injury is still controversial. Because the large bone flap operation has great damage, it may increase the severe disability and plant survival due to the reduction of mortality and increase the burden on families and society. After craniotomy and decompression, the small blood vessel or barrier damaged by the plaintiff in the adjacent or remote part of the hematoma bled again due to loss of blockage. Compared with traditional craniotomy, the effects of reducing intracranial pressure and improving the prognosis of patients need to be further explored [5]. Therefore, by analyzing the clinical data of 89 patients with severe craniocerebral injury, this study explores the effects of different surgical methods on neurological function, cerebral hemodynamic parameters, and prognosis. Furthermore, the clinical effect of large bone flap craniotomy on patients with severe craniocerebral injury is analyzed, which can provide a theoretical basis for improving the prognosis of these patients.

The article "Investigation of the Effects of Large Bone Flap Craniotomy on Cerebral Hemodynamics, Intracranial Infection Rate, and Nerve Function in Patients with Severe Craniocerebral Trauma" was retracted in 2023. Reasons: signs of a paper mill; suspected computer-generated content; unreliable results or conclusions; lack of ethics approval or compliance.

The remainder of this paper is organized as follows.  Section 2 discusses the related work, followed by the general information and methods in Section 3. The results and analysis is discussed in Section 4.  Section 5 concludes the paper with a summary.

## 2. Related Work

The injury of patients with craniocerebral trauma is related to hematoma, and the intracranial pressure can lead to the patient's disturbance of consciousness or coma [6]. The common complications of severe craniocerebral injury mainly refer to the complications of other parts except the craniocerebral injury itself. In addition, there are combined injuries with other parts, such as hemopneumothorax, intraperitoneal visceral hemorrhage, open limbs, or fractures in other parts. For severe craniocerebral injury, patients with obvious increase of intracranial pressure or combined with brain stem and hypothalamus injury are very prone to gastrointestinal bleeding within 3–10 days after injury. In addition, some patients are prone to respiratory tract infection and even severe pneumonia due to severe injury and long coma. One of the most effective methods for surgical treatment of severe craniocerebral injury is the traditional bone window craniotomy. Because the incision area is small, the vision of the operator is limited, so it will also affect the clearance of hematoma and brain tissue necrosis. However, with the development of medical technology, the surgical technique of large bone flap craniotomy is also improving and has been widely used in clinic [7, 8]. It should be noted that most studies have not reported the effects of the two operations on cerebral hemodynamic parameters and neurological function in patients with severe craniocerebral injury [9].

As a common symptom after severe craniocerebral injury, the level of intracranial pressure is usually more than four times that of normal people. Large bone flap craniotomy can improve the clearance rate of intracranial hematoma and necrotic tissue by increasing the incision length and fully exposing the intraoperative visual field. Thus, CBF and CBV can be increased [10, 11]. Hu et al. [12] showed that large bone flap craniotomy can improve the clearance rate of hematoma, increase the compensatory space of the brain, further reduce the intracranial pressure and reduce the occurrence of postoperative complications. However, some scholars have pointed out that expanding the area of bone flap resection can enhance the compensatory volume of the skull. However, due to the unique physiological function and structure of the brain, the scope of bone flap resection cannot be expanded indefinitely. Otherwise, adverse postoperative events will occur and further aggravate the disease [13].

Traditional bone flap craniotomy surgery due to bone window area is limited, lead to necrotic tissue thoroughly cleared, intracranial pressure. Mosaic is easy to make the body tissue and bone window edge position. However, large bone flap craniotomy can fully expose the anterior, middle cranial fossa, frontal lobe, parietal lobe, and other parts during the operation, which can rapidly and effectively reduce intracranial pressure. In addition, cerebral hernia can be reduced after the reduction of intracranial pressure and further reduce the occurrence of postoperative complications [14–16]. At the same time, the neurological function recovery of the large bone flap group is better than that of the control group, which can also explain the abovementioned points. Decompression of the large bone flap can accelerate blood reflux and improve the brain microcirculation of patients, so as to reduce the pressure of hematoma and thrombosis on the cerebral veins and improve the neurological function [17–19]. Large bone flap craniotomy in patients with a severe craniocerebral injury can effectively improve the survival status of prognosis, effectively reduce intracranial pressure, reduce the compression of intracranial necrotic tissue and hematoma on cerebral vessels, and improve the cerebral blood supply capacity. Therefore, it is not necessary to improve the postoperative survival rate [20, 21].

The article "Investigation of the Effects of Large Bone Flap Craniotomy on Cerebral Hemodynamics, Intracranial Infection Rate, and Nerve Function in Patients with Severe Craniocerebral Trauma" was retracted in 2023. Reasons: signs of a paper mill; suspected computer-generated content; unreliable results or conclusions; lack of ethics approval or compliance.

In this study, intracranial pressure decreased in both groups after surgical treatment. The intracranial pressure in the large bone flap group was lower than that in the control group at T2 and T3. This indicates that the large bone flap craniotomy is an ideal result to reduce intracranial pressure. In addition, the purpose of this study is to observe different cerebral hemodynamic parameters. In patients with craniocerebral trauma, CBF and CBV decreased in varying degrees due to severe brain tissue damage and insufficient blood supply [22, 23]. However, after treatment, the CBF and CBV of the two groups were improved, and the large bone flap group was better than the control group at different times after improvement. Furthermore, large bone flap craniotomy can effectively reduce intracranial pressure in a short time after operation, reduce postoperative complications, improve neurological function, and improve survival rate. It has a high clinical value in patients with severe craniocerebral injury.

## 3. General Information and Proposed Methods

### 3.1. General Information

A retrospective analysis was performed on 89 patients with severe craniocerebral trauma admitted from January 2020 to June 2021. According to different surgical methods, they were divided into a large bone flap group (*n* = 45) and control group (*n* = 44). The comparison of baseline data between groups is shown in Table 1, and there was no statistical difference in general information (all *P* < 0.05), indicating comparability. All patients included in the study signed informed consent before surgery and understood the risks associated with surgery and the possible complications after surgery. Meanwhile, the clinical data obtained in this study will only be used for research, not for other purposes.

The article "Investigation of the Effects of Large Bone Flap Craniotomy on Cerebral Hemodynamics, Intracranial Infection Rate, and Nerve Function in Patients with Severe Craniocerebral Trauma" was retracted in 2023. Reasons: signs of a paper mill; suspected computer-generated content; unreliable results or conclusions; lack of ethics approval or compliance.

Inclusion criteria are as follows: (1) meet the clinical diagnostic criteria for severe craniocerebral trauma [24]; (2) complete general information and clinical data; (3) signing informed consent and surgical consent; and (4) high treatment compliance.

Exclusion criteria are as follows: (1) persons with immune deficiency; (2) people with coagulation disorder; (3) those with a history of craniotomy; and (4) patients with mental diseases that affect the evaluation of postoperative neurological function, as shown in Table 1.

### 3.2. Proposed Methods

#### 3.2.1. Surgical Methods

The two groups were treated with tracheal intubation and general anesthesia before surgery and supine position during surgery.

The control group received conventional craniotomy decompression, which was performed as follows: a horseshoe incision was made in the temporal parietal or temporal frontal area of the patient, and the bone flap with a range of (6 × 8) cm was removed to remove the hematoma and injured lesion tissue, and hemostatic measures were taken to stop the broken blood vessels. After hemostasis, we placed the drainage tube, checked dura mater, confirmed no problem, and sutured.

In the large bone flap group, the specific steps of large bone flap craniotomy are as follows: (1) connect the zygomatic arch or external canthus with the external auditory canal, take 1 cm in front of the tragus as the starting point of the incision; (2) extend along the posterior upper part of the auricle to the apical tubercle and 2 cm beside the median line; (3) cut the subcutaneous tissue from the midline forward to the forehead hair line or between eyebrows, and the removal range is (10 × 12) Cm bone flap, suspended a circle of dura mater and cut radially; (4) fully expose the anterior and middle floor of frontal lobe, the bottom of temporal lobe and temporal pole, clear the hematoma and damaged local tissue, and take hemostatic measures to stop bleeding; and (5) after hemostasis, a drainage tube was placed to repair the artificial meninges and temporal fascia.

Both groups were treated with antibiotics, dehydration, and brain cell nutrition.

#### 3.2.2. Detection of Cerebral Hemodynamic Parameters

Cerebral blood flow (CBF), cerebral blood volume (CBV), and time to peak (TTP) were measured by CT perfusion imaging at stage T1, T2, and T3, respectively. The intracranial pressure detection probe is placed in the skull and the probe should be placed on the forehead and occipital bone. The intracranial pressure waveform is transmitted to the workstation through the sensor to monitor the changes of the patient's intracranial pressure.

The article "Investigation of the Effects of Large Bone Flap Craniotomy on Cerebral Hemodynamics, Intracranial Infection Rate, and Nerve Function in Patients with Severe Craniocerebral Trauma" was retracted in 2023. Reasons: signs of a paper mill; suspected computer-generated content; unreliable results or conclusions; lack of ethics approval or compliance.

#### 3.2.3. Assessment of Neurological Impairment (NIHSS)

The NIHSS scale is mainly used to evaluate the degree of neurological impairment of patients. It can evaluate the neurological function through a comprehensive analysis of consciousness level, gaze, visual field, upper and lower limb motor function, ataxia, and other aspects. The score range is 0 to 42, and the higher the score, the more severe the degree of neurological impairment of patients.

### 3.3. Statistical Treatment

SPSS 25.0 statistical software was used for data analysis: (1) a normality test was performed on the data first. If the data followed normal distribution and homogeneity of variance, they were represented by mean ± standard deviation. Paired sample *t* was used for test within the group, variance comparison was used between groups, and F test was performed for comparison between multiple groups; (2) counting data and percentage representation, *χ*^2^ test; and (3) the Kaplan–Meier survival curve was used to observe the postoperative survival rate of patients in the two groups, and the follow-up period was up to December 2021. *P* < 0.05 indicated significant difference.

## 4. Results and Analysis

### 4.1. Observation of Cerebral Hemodynamic Indexes

Preoperative differences in cerebral hemodynamics and intracranial pressure were not significant (*P* > 0.05), postoperative TTP and intracranial pressure were decreased in the two groups, and the large bone flap group was lower than the control group at T2 and T3 stages. CBV and CBF increased in both groups after surgery, and T2 and T3 in the large flap group were higher than the control group (both *P* < 0.05), as shown in Table 2 and Figure 1. The symbol “^*∗*^” means that compared with T1, ^*∗*^*P* < 0.05; # indicates that compared with T2, #*P* < 0.05.

### 4.2. Incidence of Postoperative Intracranial Infection

The incidence of postoperative intracranial infection in the large flap group was significantly lower than that in the control group, and the incidence of postoperative total adverse events was also lower than that in the control group (*P* < 0.05), as shown in Table 3.

### 4.3. Neurological Function Assessment

Compared with before surgery, the neurological function of both groups recovered after surgery, and the improvement effect of the large flap group was significantly better than that of the control group (*P* < 0.05), as shown in Table 4.

### 4.4. Survival Rate Comparison

The Kaplan–Meier survival curve showed that the postoperative survival rate of the large flap group was significantly higher than that of the control group (*χ*^2^ = 5.145, *P*=0.023), as shown in Figure 2.

The article "Investigation of the Effects of Large Bone Flap Craniotomy on Cerebral Hemodynamics, Intracranial Infection Rate, and Nerve Function in Patients with Severe Craniocerebral Trauma" was retracted in 2023. Reasons: signs of a paper mill; suspected computer-generated content; unreliable results or conclusions; lack of ethics approval or compliance.

### 4.5. Comparison of Plant States

Although there was no significant difference in the number of postoperative cases of vegetative states between the two groups, the number of cases of vegetative states in the large bone flap group was slightly lower than that in the control group, as shown in Table 5.

## 5. Conclusions

In this study, the effects of standard large bone flap craniotomy on cerebral hemodynamic indexes, incidence of postoperative intracranial infection, and neurological function in patients with severe craniocerebral trauma are investigated. 89 patients with severe craniocerebral trauma admitted from January 2020 to June 2021 are analyzed retrospectively. From the experimental results, it is clearly evident that the two surgical methods have certain clinical efficacy in the treatment of patients with severe craniocerebral trauma. Comparatively, the large craniotomy can further improve brain blood supply and improve neurological function recovery. Also, it can obtain low incidence of postoperative adverse reactions and intracranial infection. In the future work, we will further explore the rehabilitation nursing after the operation of severe craniocerebral injury and pay attention on how to accelerate the recovery progress of patients and reduce the postoperative mortality.

## Figures and Tables

**Figure 1:** Observation of cerebral hemodynamic indexes: (a) CBF; (b) CBV; (c) TTP; (d) intracranial pressure.

**Figure 2:** Survival rate comparison.

**Table 1:** General information for comparison.

Group	Control group (*n* = 44)	Large bone flap group (*n* = 45)	t/*x*2	*P*
*Gender*			0.280	0.597
Man	21 (47.73%)	24 (53.33%)		
Woman	23 (52.27%)	21 (46.67%)		
Age	45.04 ± 7.74	44.56 ± 7.49	0.297	0.767
BMI (kg/m2)	23.26 ± 2.21	23.66 ± 2.16	−0.864	0.390
Preoperative GCS score	5.02 ± 1.23	5.05 ± 1.21	−0.116	0.908
Injury cause			0.321	0.642
Falling	11 (25.00%)	13 (28.89%)		
Car accident	18 (40.91%)	16 (35.56%)		
Blow hurt	9 (20.45%)	11 (24.44%)		
Others	6 (13.64%)	5 (11.11%)		

**Table 2:** Comparison of cerebral hemodynamic parameters and intracranial pressure.

Group	Control group (*n* = 44)	Large bone flap group (*n* = 45)	*t*	*P*
CBF (ml/(100 g ^*∗*^ min))				
T1	22.36 ± 5.34	22.68 ± 5.27	−0.285	0.777
T2	27.95 ± 5.57^*∗*^	37.52 ± 6.42^*∗*^	−7.504	<0.001
T3	32.15 ± 5.83^*∗*#^	38.09 ± 6.38^*∗*^	−4.582	<0.001
CBV (ml/100g)				
T1	1.03 ± 0.21	1.02 ± 0.23	0.214	0.831
T2	1.41 ± 0.34^*∗*^	2.13 ± 0.53^*∗*^	−7.609	<0.001
T3	1.60 ± 0.39^*∗*#^	2.27 ± 0.56^*∗*^	−6.536	<0.001
TTP (s)				
T1	23.32 ± 2.03	23.24 ± 2.04	0.185	0.853
T2	19.01 ± 1.74^*∗*^	15.98 ± 1.67^*∗*^	8.382	<0.001
T3	17.67 ± 1.68^*∗*#^	16.04 ± 1.73^*∗*^	4.508	<0.001
Intracranial pressure (mmHg)				
T1	32.34 ± 4.21	32.27 ± 4.15	0.079	0.937
T2	26.50 ± 3.83^*∗*^	24.33 ± 3.45^*∗*^	2.810	0.006
T3	22.72 ± 3.35^*∗*#^	17.84 ± 2.75^*∗*#^	7.519	<0.001

The article "Investigation of the Effects of Large Bone Flap Craniotomy on Cerebral Hemodynamics, Intracranial Infection Rate, and Nerve Function in Patients with Severe Craniocerebral Trauma" was retracted in 2023. Reasons: signs of a paper mill; suspected computer-generated content; unreliable results or conclusions; lack of ethics approval or compliance.

**Table 3:** Incidence of postoperative intracranial infection.

Group	Number	Intracranial infection	Cerebral infarction	Cerebrospinal fluid leaking	Traumatic encephalocele	Total complication
Control group	44	8 (18.18%)	7 (15.91%)	3 (6.82%)	4 (9.09%)	22 (50.00%)
Large bone flap group	45	2 (4.44%)	3 (6.67%)	2 (4.44%)	2 (4.44%)	9 (20.00%)
*χ * ^2^		4.210	1.905	0.236	0.764	8.821
*P*		0.040	0.167	0.627	0.382	0.003

**Table 4:** Neurological function assessment.

Group	Number	Preoperative	1 month after surgery	*t*	*P*
Control group	44	33.15 ± 3.34	26.27 ± 3.20	9.866	<0.001
Large bone flap group	45	33.22 ± 3.29	21.91 ± 2.87	17.378	<0.001
T		−0.100	6.770		
*P*		0.921	<0.001		

**Table 5:** Contrast of plant states.

Group	Number	Vegetative state
Control group	44	8 (18.18%)
Large bone flap group	45	3 (6.67%)
*χ* ^2^		4.210
*P*		0.099

## Data Availability

The simulation experiment data used to support the findings of this study are available from the corresponding author upon request.
